# Increasing Strawberry Fruit Sensorial and Nutritional Quality Using Wild and Cultivated Germplasm

**DOI:** 10.1371/journal.pone.0046470

**Published:** 2012-10-03

**Authors:** Jacopo Diamanti, Franco Capocasa, Francesca Balducci, Maurizio Battino, Jim Hancock, Bruno Mezzetti

**Affiliations:** 1 Dipartimento di Scienze Agrarie, Alimentari e Ambientali, Università Politecnica delle Marche, Ancona, Italy; 2 Dipartimento di Scienze Cliniche Specialistiche ed Odontostomatologiche, Università Politecnica delle Marche, Ancona, Italy; 3 Department of Horticulture, Michigan State University, East Lansing, Michigan, United States of America; Washington State University, United States of America

## Abstract

**Background:**

Increasing antioxidant levels in fruit through breeding is an important option to support higher antioxidant intake particularly when fruit consumption is low. Indeed, if nutritional components are also combined with a high standard of sensorial fruit quality, the perspective for consumer health can be further improved by encouraging more fruit consumption. Wild species are valued by strawberry breeders as sources of novel traits, especially for pest resistance and abiotic stress tolerance. Furthermore, previous investigations have shown improvements in fruit nutritional quality in breeding material that originated from *Fragaria virginiana* ssp. *glauca* (FVG) inter-species crosses. Recently, commercial varieties of strawberries have also shown interesting variability in fruit nutritional quality.

**Results:**

Strawberry fruit sensorial and nutritional qualities generated by *Fragaria* inter-species and intra-species crosses were evaluated on 78 offspring derived from 8 families: two that originated from *F. × ananassa* intra-species crossing; three from back-crossing of F1– FVG × *F. × ananassa*; and three from back-crossing of BC1– FVG × *F. × ananassa*. The genetic variability from the three types of cross combinations was analyzed by calculation of the correlations among the fruit sensorial and nutritional parameters. The results obtained show that two subsequent back-crossing generations from an inter-species crossing combination with *F. virginiana* ssp. *glauca* provides useful improvement of the fruit nutritional and sensorial qualities that is combined with agronomic standards that are close to those requested at the commercial level. Improvements of these traits can also be achieved by programming *F. × ananassa* intra-species crosses and producing progeny with productivity traits more similar to those of the commercial cultivars.

**Conclusions:**

The two types of combination programs (inter-species back-crosses, and intra-species crosses) can be used to improve strawberry nutritional quality.

## Introduction

Greater consumption of fruit and vegetables is considered as one way of increasing the intake of antioxidants, and like other berries, strawberry represents one of the most important sources of bioactive compounds with high antioxidant capacity [1]–[6]. Accordingly, an increase in the consumption of berries richer in ‘healthy compounds’ is seen as an appropriate strategy for improving human health.

Increasing the antioxidant levels in fruit through breeding and/or biotechnology is an important option to maintain a higher antioxidant intake, particularly when fruit consumption is low. Indeed, if nutritional bioactive components are combined with a high standard of sensorial fruit quality, consumer fruit consumption can be encouraged, with much greater positive health effects [3], as would be the case for strawberry fruit [7].

The breeding of more nutritious, better-tasting cultivars can be successful if the variability and heritability of the bioactive compounds, which is defined as the total antioxidant capacity (TAC), indicate the possibility of achieving breeding progress. It is well know that the availability of genetic diversity within compatible species of any given crop will enhance the extent of any improvement [8]. The biotechnological approach is also an option to supplement this improvement, through modifications of specific biosynthetic pathways [9]. However, the success of both breeding and biotech approaches is dependent on deep knowledge of the sources of the most useful wild and cultivated genetic diversity to be used in genetic and genomic studies.

The effect of genotype on the nutritional quality of strawberry is well known [10]–[13]. The levels of antioxidants and the TAC in strawberry extracts from whole fruits vary considerably among genotypes [4], [12], [14], although few genotypes have been well characterized for these important features. Furthermore, limited knowledge is available on the possibility of improving strawberry nutritional traits by breeding [15]–[16]. Some results have been obtained for blueberries and raspberries, with a moderate heritability for TAC, total phenols content (TPH) and anthocyanins content (ACY) demonstrated [17]–[21].

Accessions of the progenitor wild species are valued by strawberry breeders as sources of novel traits, and especially for pest resistance and abiotic stress tolerance [22]. Furthermore, previous investigations [4], [5], [15], [16] have shown improvements in fruit nutritional quality in breeding material that originated from *Fragaria virginiana* ssp. *glauca* (FVG) in inter-species crosses. This result is supported by a study carried out by Wang *et al.* [14] that showed that the fruit of *F. virginiana* accessions have significantly higher TAC, TPH, and total ACY than the fruit from different lines of *F. chiloensis* and *F. × ananassa*.

Since 2006, a breeding program based on the evaluation and comparison of different populations of *F. × ananassa* crosses and FVG inter-species back-crosses has been conducted by the *Università Politecnica delle Marche*, with the objective being to generate new selections with increased fruit nutritional quality.

With the aim of studying strawberry fruit sensory and nutritional quality generated by *Fragaria* inter-species and intra-species crosses, 78 offspring derived from 8 families were evaluated, two originating from *F. × ananassa* intra-species crosses; three from back-crossing of F1– FVG × *F. × ananassa*; and three from back-crossing of BC1– FVG × *F. × ananassa* (Figure 1). The selection AN94,414,52 (F1 FVG) used in the breeding program was originated by the inter-species cross of *F. virginiana* ssp. g*lauca* “FVG22” × *F. × ananassa* selection 91,143,5. FVG22 is a clone of *F. virginiana* ssp. g*lauca* that is maintained in the National Clonal Germplasm Repository in Corvallis (OR, USA), while the *F. × ananassa* selection 91,143,5 originated from the breeding program of the Italian Experimental Agriculture Research Council, Forli Fruit Research unit (CRA-FRF, Italy).

**Figure 1:** Crossing combination scheme. Scheme of the crossing combinations, including *F. × ananassa* and *F. virginiana glauca* back-crossing, and *F. × ananassa* intra-species crossing.

Fruit sensorial and nutritional parameters of all of the offspring were evaluated in 2009 from single seedling plants, and in 2010 on vegetatively propagated selections. For both years, all of the offspring and the corresponding parents were evaluated for their fruit nutritional qualities (fruit TAC, TPH and ACY), while in the second year, they were evaluated for their production (fruit weight and total plant production, commercial, misshapen, undersized and rotten fruit production, per plant) and sensorial (fruit firmness, color, solid soluble [SS] content and total acidity [TA]) parameters.

The genetic variability that originated from the three types of cross-combinations (BC1 back-cross, BC2 back-cross, and intra-species cross) was analyzed by correlating fruit sensorial and nutritional parameters. With such an analysis, we were able to evaluate the relative effects of intra-species and inter-species back-cross populations.

## Results

Fruit nutritional and sensorial parameters of the different breeding populations were evaluated by two-way nested ANOVA, which revealed significant differences between the inter-species back-crosses and the intra-species crosses (Table 1).

**Table 1:** Two-way nested ANOVA for the type of cross combination and the individual BC1, BC2 and intra-species populations for the fruit sensorial and nutritional parameters.

Factor	DF	SS content (°Brix)		TA (meq NaOH/100 g FW)		Firmness (g)		L*		Chroma		TAC (mmol TE/kg FW)		TPH (mg GA/kg FW)		ACY (mg PEL-3-GLU/kg FW)	
		MS	F	MS	F	MS	F	MS	F	MS	F	MS	F	MS	F	MS	F
Type of cross	2	7,.1	10.9	52.8	16.1	21363	9,7	66.2	17.4	87.3	8.8	338.1	65.1	299300	3.6	103216	9.3
Error	7	0.7		3.3		2195		3.8		9.9		5.2		83518		11076	
BC1 POP	2	1.1	1.5	7.2	1.8	1768.0	0.8	1.7	0.4	12.4	1.0	138.4	16.5	198108.5	1.4	12373.1	1.1
Error	28	0.7		4.0		2139.4		4.2		11.8		8.4		144708.2		11218.8	
BC2 POP	2	1.5	2.5	17.9	5.6	1491.7	1.0	17.5	5.8	36.3	4.2	313.6	81.2	347355.1	12.4	10471.7	0.9
Error	22	0.6		3.2		1442.0		3.0		8.6		3.9		27991.4		11191.3	
IS POP	1	0.5	0.8	13.7	8.3	5873.3	2.4	79.6	16.7	158.2	16.6	4.7	2.5	546376.7	9.7	57935.4	5.4
Error	18	0.7		1.7		2449.8		4.8		9.5		1.9		56198.9		10712.1	

ANOVA analysis was calculated between the types of crossing and within each cross combination. For each factor of analysis, the degree of freedom (DF), mean square (MS) and F value (F) for the sensorial and nutritional parameters were evaluated and are reported. IS, intra-species; POP, population.

SS content, TA, TAC, TPH and ACY were significantly higher in the BC1 and BC2 back-crossed populations that contained genes from *Fragaria virginiana* ssp *glauca* (Table 2) than in the *F. × ananassa* intra-species crosses, while the intra-species crosses were firmer and more darkly colored (Table 2). For all of the parameters examined, there were no significant differences between the BC1 and BC2 back-crosses, although the individual populations were significantly different.

**Table 2:** Fruit sensorial and nutritional parameters of the clonal populations of selected seedlings for each of the individual cross combinations within the BC1 and BC2 back-crosses and the intra-species cross populations.

Type of cross	Cross code	SS content (°Brix)	TA (meq NaOH/100 g FW)	Firmness (g)	Chroma	L*	TAC (mmol TE/kg FW)	TPH (mg GA/kg FW)	ACY (mg PEL-3-GLU/kg FW)
BC1	AN07,003	9.32 ns (0.24)	11.75 b (0.42)	338.85 ns (9.86)	45.55 ns (0.47)	34.49 ns (0.39)	20.91 b (0.53)	1604.53 b (70.54)	494.6 a (19.89)
BC1	AN07,004	9.07 ns (0.23)	13.37 a (0.4)	321.51 ns (9.57)	44.29 ns (0.46)	34.41 ns (0.37)	23.54 a (0.52)	1875.13 a (68.49)	429.08 b (17.37)
BC1	AN07,005	9.79 ns (0.24)	12.01 ab (0.42)	349.33 ns (9.86)	43.51 ns (0.47)	33.85 ns (0.39)	16.17 c (0.53)	1650.77 ab (70.54)	457.77 ab (17.89)
BC2	AN07,006	8.93 ns (0.22)	12.48 b (0.39)	341.07 ns (0.37)	42.88 ab (0.45)	35.60 a (8.98)	22.88 b (0.4)	1558.72 b (37.34)	498.49 ns (21.39)
BC2	AN07,215	9.44 ns (0.26)	15.38 a (0.45)	312.41 ns (0.42)	44.81 a (0.52)	35.54 a (10.31)	27.21 a (0.46)	1964.33 a (42.87)	446.10 ns (24.55)
BC2	AN07,216	8.53 ns (0.22)	12.71 b (0.39)	336.47 ns (0.36)	41.09 b (0.44)	33.62 b (8.83)	15.12 c (0.39)	1657.34 b (36.71)	505.69 ns (21.03)
IS	AN07,007	8.42 ns (0.23)	11.4 a (0.31)	363.58 ns (10.88)	49.65 a (0.59)	39.69 a (0.43)	14.78 ns (0.43)	1690.76 a (39.06)	288.94 b (16.33)
IS	AN07.009	8.78 ns (0.25)	9.74 b (0.29)	398.71 ns (10.20)	44.03 b (0.54)	35.73 b (0.46)	13.80 ns (0.40)	1363.16 b (34.63)	393.35 a (17.64)

Data are means and standard errors (SE) of the offspring selections for each family. Means followed by different letters are significantly different. SNK Test P≤0.05. IS, intra-species.

### Selections of the BC1 Populations

The two-way nested ANOVA evaluated for the BC1 back-cross populations showed significant differences for fruit TA, TAC, TPH and ACY, but not for SS content, firmness, Chroma and L* (Table 1).

The highest mean values of the fruit TA were seen for AN07,004 and AN07,005, while the AN07,003 cross-combination showed a significantly lower TA than for AN07,004, although not a significantly different TA than for AN07,005 (Table 2). The highest fruit TAC was seen for the fruit of AN07,004, while the lowest was for the fruit of AN07,005; these TACs were significantly different. Population AN07,004 also showed the highest fruit TPH, which was significantly different from the AN07,003 back-cross population with the lowest TPH (Table 2).

In contrast to these results, population AN07,003 showed the highest fruit ACY, which was significantly higher than for AN07,004 (Table 2).

The BC1 populations also differed significantly in their plant production parameters. Indeed, AN07,004 had the highest mean for fruit weight and commercial production, and the lowest for misshapen fruit per plant (Table 3). The lowest mean fruit weight was seen for AN07,003, while the lowest commercial production was for AN07,005. The lowest amount of rotted fruit was seen for BC1 AN07,004 (Table 3).

**Table 3:** Plant production parameters of the selections from the BC1 and BC2 back-cross and the intra-species cross populations.

Type of cross	Cross code	Fruit weight (g/20 fruits)	Misshapen fruit (g/plant)	Undersized fruit (g/plant)	Rotten fruit (g/plant)	Commercial production (g/plant)	Total production (g/plant)
BC1	AN07,003	11.7 (0.6)	18.5 (5.4)	110.5 (19.1)	78.8 (16.6)	349.0 (26.7)	556.8 (39.2)
BC1	AN07,004	13.9 (1.0)	10.4 (2.9)	116.7 (20.2)	48.4 (7.8)	356.7 (52.7)	532.1 (54.0)
BC1	AN07,005	12.9 (0.1)	15.0 (3.5)	190.8 (38.7)	62.4 (12)	300.5 (41.2)	568.6 (67.9)
BC2	AN07,006	14.4 (0.8)	15.1 (3.9)	162.1 (21.9)	77.2 (7.7)	401.6 (29.3)	656.1 (41.9)
BC2	AN07,215	13.6 (0.5)	3.9 (1.5)	97.8 (31.3)	135.6 (34.8)	265.6 (35.3)	502.2 (40.1)
BC2	AN07,216	14.7 (0.9)	10.7 (4.1)	110.5 (28.2)	51.1 (11.5)	376.3 (48.9)	548.6 (76.3)
IS	AN07,007	16.3 (1.0)	27.5 (5.1)	103.0 (11.5)	182.0 (32)	464.3 (38.9)	776.8 (57.7)
IS	AN07,009	18.0 (0.6)	22.1 (5.7)	76.3 (14.8)	190.9 (36.4)	431.1 (38.2)	720.4 (80.3)

Data are means and standard errors (SE) of the offspring selections for each family.

Fruit sensorial and nutritional parameters of the BC1 populations had different levels of correlation (Table 4). Fruit TA was negatively correlated with fruit SS content (−0.24), firmness (−0.50) and ACY (−0.30). A high negative correlation was also seen between fruit firmness and TAC (−0.34). The Chroma index had a high negative correlation with TAC (−0.29) and ACY (−0.46). Finally, L* grade showed a high negative correlation with fruit ACY (−0.47) (Table 4).

**Table 4:** Pearson’s correlation matrix of the fruit sensorial and nutritional parameters for type of crossing evaluated on clonal populations of selected seedling.

BC1 populations		SS content	TA	Firmness	Chroma	L*	TAC	TPH
	SS content	–						
	TA	−0.24**	–					
	Firmness	0.03	−0.50^$^	–				
	Chroma	0.03	−0.08	0.05	–			
	L*	0.16	−0.11	−0.04	0.83^$^	–		
	TAC	0.02	0.06	−0.34^$^	−0.29^$^	−0.14	–	
	TPH	0.06	−0.12	−0.15	−0.10	−0.07	0.46^$^	–
	ACY	0.26**	−0.30**	−0.07	−0.46^$^	−0.47^$^	0.33^$^	0.18
**BC2 populations**	SS content	–						
	TA	0.18	–					
	Firmness	−0.22*	−0.24*	–				
	Chroma	−0.02	0.01	−0.09	–			
	L*	0.04	0.06	−0.26*	0.82^$^	–		
	TAC	0.29**	0.45^$^	−0.21*	0.15	0.20*	–	
	TPH	0.29**	0.44^$^	−0.17	0.08	0.15	0.47^$^	–
	ACY	0.02	0.04	0.24*	−0.62^$^	−0.65^$^	0.04	0.07
**Intra-species cross populations**	SS	–						
	TA	−0.16	–					
	Firmness	−0.06	−0.19	–				
	Chroma	0.21	0.28*	−0.48^$^	–			
	L*	0.26*	0.12	−0.44^$^	0.75^$^	–		
	TAC	0.03	0.27*	−0.05	0.07	0.15	–	
	TPH	0.02	0.34**	−0.10	0.23*	0.30**	0.83^$^	–
	ACY	−0.08	−0.22*	0.28*	−0.64^$^	−0.53^$^	0.37^$^	0.18

* , **, ^$^ correlation levels significant at p≤0.05; p≤0.01; p≤0.001 respectively.

Positive correlations were seen between SS content and fruit ACY (0.26), Chroma index and L* grade (0.83), and fruit TAC and TPH (0.46) and ACY (0.33) (Table 4).

These data show the positive effects of using *F. virginiana glauca* in strawberry breeding, in terms of improving the fruit nutritional parameters, although there was a negative effect on fruit sensorial parameters, as shown by the correlation matrix for the BC1 FVG back-crosses. Indeed, the increase in fruit nutritional parameters was associated with a large increase in fruit TA, which was linked with a decrease in fruit SS content, firmness and ACY. In particular, fruit TAC was negatively correlated with fruit firmness and Chroma index. This indicates that in BC1 progenies, the higher content of bioactive compounds that determine the fruit TAC is associated with negative effects on fruit firmness, color (darker fruit) and ACY. The correlation matrix of the same BC1 progenies reveals negative correlation between ACY and both colorimetric parameters, while in the BC1 population, ACY was positively correlated with an increase in fruit SS content. Among the nutritional parameters, the positive correlations between fruit TAC and TPH, and fruit TAC and ACY were consistent with what was reported by Scalzo et al. (2005).

Principal component analysis (PCA) bi-plots of the BC1 families showed strong associations between the TAC and TPH nutritional parameters for AN07,004, and in particular for AN07,004,51 and AN07,004,54 (Figure 2b), confirming the data for the nutritional parameters in Table 4. AN07,003 showed the highest fruit ACY (Table 2) and PCA analysis confirmed this trend (Figure 2b). The PCA bi-plots combining the data of the fruit TAC, TPH, ACY, and weight, and the commercial production of the selections and corresponding parents of the BC1 populations (Figure 2a, vector distribution plot; Figure 2b, case distribution plot), highlight the selections AN07,004,51, AN07,004,52, AN04,007,54 and AN07,003,60 for their positions in the upper right-hand section of the plot, corresponding to high values of the fruit ACY, TPH and TAC variables. Thus, these selections have the highest fruit nutritional value, although they still have some deficiencies in fruit fresh weight and the levels of commercial production. Conversely, selections AN07,004,57 and AN07,005,58 are located in the upper left-hand quadrant of the plot, located towards the vectors of fruit weight and commercial production. All of the other offspring are located between the positions of the parents, which are in the central area of the plot. The male parents (cv. Alba and Clery, selection Romina) are situated on the left-hand side of the plot, again, corresponding to the vectors of fruit weight and commercial production, while the common female parent, the F1 selection AN94,414,52, is located on the right-hand side of the plot, corresponding to the vectors of fruit TAC, TPH and ACY. This confirms the offspring improvement in fruit size and plant production with regard to the FVG mid-parent [22].

**Figure 2:** Principal component analysis. Bi-plot of the fruit weight, commercial production, TAC, TPH and ACY parameters of the selections and their corresponding parents, of the BC1 back-cross populations. Factor 1 and Factor 2 explain 67.57% of the data variation. a: Variable vector distributions; b: Case distributions. The seedlings reported in the PCA are identified only with the codes related to the cross combinations and the progressive seedling numbering.

The PCA bi-plots of the BC1 families for fruit sensorial parameters (SS content, TA) combined with fruit weight and commercial production variables (Figure 3a) locates most of the selections towards the SS content vector instead of the fruit weight and commercial production vectors, revealing an improvement in the sensorial quality of the progenies, with respect to their parents (Figure 3b). With all three of the families more towards the SS content vector, AN07,003,60 is the selection that is most oriented towards the fruit SS content vector.

**Figure 3:** Principal component analysis. Bi-plot of fruit weight and commercial production *versus* SS content and TA for the offspring and parents of the BC1 back-cross populations. Factor 1 and Factor 2 explain 80.46% of the data variation. a: Variable vector distributions; b: Case distributions. The seedlings reported in the PCA are identified only with the codes related to the cross combinations and the progressive seedling numbering.

In the PCA bi-plots of the BC1 families for Chroma index, fruit ACY and TPH (Figure 4a, vector distributions), most of the offspring and parents are distributed in the left-hand central area of the plot, where the Chroma index vector is located (Figure 4b, case distributions). The only exceptions are selections AN07,003,60 and AN07,004,54: AN07,003,60 is located on the right-hand side of the plot, towards the vector of the fruit ACY variable, and AN07,004,54 is located in the upper right-hand quadrant, in the direction of the fruit TPH.

**Figure 4:** Principal component analysis. Bi-plot of the ACY, TPH and Chroma index components for the offspring and the parents of the BC1 back-cross populations. Factor 1 and Factor 2 explain 87.25% of the data variation. a: Variable vector distributions; b: Case distributions. The seedlings reported in the PCA are identified only with the codes related to the cross combinations and the progressive seedling numbering.

These data on the fruit sensorial and nutritional parameters demonstrate the importance of using the F1 FVG parent in the breeding, as it positively influences the fruit nutritional characteristics of the progeny seedlings.

### Selections of the BC2 Populations

The ANOVA analysis of the BC2 population in 2010 showed significant differences for fruit TA, Chroma index, L* grade, TAC and TPH, while there were no significant differences for fruit SS content, firmness and ACY (Table 1).

The significant highest mean values for fruit TA, Chroma index, TAC and TPH were seen for AN07,215, while the significant highest values for SS content and L* were in AN07,006 (Table 2). Fruit firmness and ACY did not show significant differences among the BC2 populations; however, the lowest fruit TA, Chroma, L* and TAC were seen in AN07,216 (Table 2).

The highest means for fruit weight and commercial production were seen in the AN07,216 and AN07,006 populations, although these also had the highest levels of misshapen and undersized fruit per plant (Table 3). The lowest mean commercial production was seen for AN07,215, together with the lowest level of misshapen and undersized fruit production per plant, although also with the highest value for rotten fruit production (Table 3). Few misshapen fruit were seen in the BC2 populations, in comparison with the intra-species cross population (Table 3).

The Pearson matrix for the fruit of the BC2 populations showed a number of negative correlations among the various sensorial and nutritional parameters (Table 4). Indeed, significant negative correlations were seen between fruit firmness and fruit SS content (−0.22), TA (−0.24), L* grade (−0.26) and fruit antioxidant capacity (−0.21). Most significantly, negative correlations were seen between fruit ACY and Chroma index (−0.62) and L* grade (−0.65) (Table 4).

Significant positive correlations were seen between TA and fruit TAC (0.45), TA and TPH (0.44), fruit TAC and TPH (0.47), and Chroma index and L* grade (0.82); also, stronger significant positive correlations were seen between SS content and TAC (0.29), and between SS content and TPH (0.29). Finally, firmness and ACY were positively correlated (0.24) (Table 4).

The results from the correlation matrix of the BC2 families show that in moving ahead by one back-cross generation there is a substantial improvement, seen as favorable correlations between sensorial and nutritional parameters. Indeed, in the BC2 populations, high fruit TAC and TPH content correspond to an increase in the fruit SS content and TA, and an increase in TAC corresponds to an increase in fruit brightness (L*) (Tables 2, 4). There are still some negative correlations, mainly for fruit firmness, which is negatively correlated with SS content, TA, L* grade and fruit TAC. So, highlighting these effects, a second back-cross generation can have positive effects for the improvement of fruit sensorial (SS content, TA, and L*) and nutritional (TAC) quality, but not of fruit firmness (Table 4). Negative correlations also remain between the fruit color parameters and ACY; indeed, in the BC2 families, high fruit ACY corresponds to a darker and more opaque fruit (Tables 2, 4).

The PCA bi-plots of fruit TAC, TPH, ACY, fruit weight and plant commercial production for the offspring and parents of these BC2 back-cross combinations (male parents: Clery, Romina and AN03,338,56; female parent: AN00,239,55) (Figure 5a) show a unique distribution for each cross combination; indeed, the seedlings of AN07,215 were almost all located in the lower right-hand quadrant of the plot, where the vectors for the fruit TAC and TPH variables are seen, in particular for the selections AN07,215,55 and AN07,215,57 (Figure 5b). The other two cross combinations are located mainly on the mid left-hand side of the plot (Figure 5b), where the vector for plant commercial production is located (Figure 5a), showing their lower affinity for the nutritional parameters. The selection AN07,216,60 here deserves special attention, as it is located in the upper right-hand quadrant where the vector for fruit ACY is positioned (Figure 4a), together with the female parent of the BC1 selection AN00,239,55.

**Figure 5:** Principal component analysis. Bi-plot of the fruit weight, commercial production, TAC, TPH and ACY parameters of the selections and the corresponding parents of the BC2 back-cross populations. Factor 1 and Factor 2 explain 67.18% of the data variation. a: Variable vector distributions; b: Case distributions. The seedlings reported in the PCA are identified only with the codes related to the cross combinations and the progressive seedling numbering.

The PCA plots for fruit sensorial parameters (SS content, TA) and productive parameters (fruit weight, commercial production) (Figure 6a) show wider distributions of the offspring for the cases plot (Figure 6b), in the offspring that are characterized by higher sensorial parameters and the offspring that are characterized by higher productive parameters.

**Figure 6:** Principal component analysis. Bi-plot of the fruit weight, commercial production, TA and SS content parameters of the selections and the corresponding parents of the BC2 back-cross populations. Factor 1 and Factor 2 explain 78.66% of the data variation. a: Variable vector distributions; b: Case distributions. The seedlings reported in the PCA are identified only with the codes related to the cross combinations and the progressive seedling numbering.

The selections AN07,215,55 and AN07,215,53 are in the lower left-hand quadrant of the plot (Figure 6b), where the SS content and TA vectors are located (Figure 6a). The selections AN07,006,62 and AN07,216,55 and the male parents (Clery and AN03,338,56) (Figure 6b) are located in the lower right-hand quadrant of the plot, showing more affinity with the fruit weight and commercial production vectors (Figure 6a).

The other selections of BC2 are positioned in the central area of the plot, or in the opposite quadrants from where the vectors are located. From this distribution, it can be noted that most of the BC2 offspring are more oriented towards the commercial production and fruit weight vectors, in comparison with the BC1 parent AN00,239,55 (Figure 6b). This confirms the greater improvement of this trait in the BC2 genotypes than in their FVG parent [22].

The PCA plot for the fruit Chroma index, TPH and ACY variables (Figure 7a) shows the distribution of the offspring (Figure 7b) around the central area of the plot, with only the selection AN07,215,55 differing from the others; indeed, it is located in the lower left-hand quadrant of the plot (Figure 7b), where the TPH vector is located. The location of the female parent AN00,239,55 is in the lower right-hand quadrant and the location of the male parent AN03,338,56 is in mid-left-hand area of the plot (Figure 7b), following the orientations of the ACY vector and the Chroma index vector, respectively (Figure 7b).

**Figure 7:** Principal component analysis. Bi-plot of the Chroma, TPH and ACY parameters of the selections and the corresponding parents of the BC2 back-cross populations. Factor 1 and Factor 2 explain 90.87% of the data variation. a: Variable vector distributions; b: Case distributions. The seedlings reported in the PCA are identified only with the codes related to the cross combinations and the progressive seedling numbering.

The offspring AN07,215,55 showed high affinity for fruit nutritional quality (Figure 5b), and the PCA bi-plot also revealed its high fruit sensorial quality (Figure 6b), which indicates a good equilibrium between fruit SS content and TA. Also, the other offspring of the AN07,215 back-cross population showed a good combination of fruit nutritional (Figure 5b) and sensorial (Figure 6b) qualities, with respect to the other BC2 populations. These selections can be considered as an important improvement from the original FVG inter-species cross combination, and to be very close to the characteristics now requested for a commercial variety.

### Selections from the Intra-species Crosses

The selections from the intra-species cross populations evaluated in 2010 differed significantly for fruit TA, Chroma index, brightness (L*), TPH and ACY, while the SS content, fruit firmness and TAC remained more stable within the populations (Table 1) and showed no significant differences.

The intra-species cross population AN07,007 (Romina × AN03,338,56) showed the most significant values for fruit TA, Chroma index, brightness (L*) and fruit TPH, while the highest fruit firmness and ACY were seen for the AN07,009 intra-species cross combination (Romina × Clery) (Table 2).

For the production parameters, the highest fruit weight was seen for AN07,009, which also had the lowest values for undersized and misshapen fruit per plant (Table 3), while AN07,007 showed the highest values of commercial production and total production (Table 3). The rotten fruit per plant were remarkable for both of these cross combinations, as this was almost half of that seen for the commercial production (Table 3).

For the Pearson’s correlations, the Chroma index showed a high level of negative correlation with firmness (−0.48) and fruit ACY (−0.64), and even the L* grade showed high negative correlation with fruit firmness (−0.44) and ACY (−0.53). Finally, negative correlation was also seen between fruit TA and ACY (−0.22) (Table 4).

Positive correlations were seen for fruit TA and Chroma index (0.28), TAC (0.27) and TPH (0.34). Fruit TPH also showed positive correlation with Chroma index (0.23) and L* grade (0.30), and high positive correlation with TAC (0.83). Fruit ACY also shown positive correlation with firmness (0.28) and high correlation with fruit TAC (0.37). Finally, fruit SS content showed positive correlation with L* grade (0.26) (Table 4).

For the intra-species cross populations, positive correlations were seen between the fruit sensorial TA and Chroma index parameters and the TAC and TPH nutritional parameters (Table 4). AN07,007 had the highest TA, Chroma index, TPH and TAC, even if the TAC was not significantly different from that detected for fruit of the AN07,009 family (Table 2). In addition, positive correlation was seen for TPH and both of the colorimetric parameters, for both families, even if the fruits of the AN07,007 cross combination showed significantly higher TPH content, Chroma index and L* grade, in comparison with the fruit of AN07,009 (Table 2). In both of these cross combinations, Romina was used as the common male parent (Table 5). Romina is a new variety that was released by the *Università Politecnica delle Marche*, and it is characterized by improved fruit sensorial and nutritional quality. It was crossed with the selection AN03,338,56 from the University breeding program, which was chosen because of its interesting sensorial and nutritional parameters, and with Clery, a well-know commercial variety on the European Union market. The differences detected for these two intra-species families reveal the influence of the Romina genetic background in the production of a high combination of fruit sensorial and nutritional parameters, and indicate that these values can be improved even more if further genetic material identified for additional improved fruit sensorial and nutritional values can be used.

**Table 5:** The families with the corresponding cross and back-cross (BC) combination, as used in the present study.

Families		Progenitors			N° of offspring	Type of cross
		Mother		Father		
A	AN07,003	AN94,414,52	×	Romina	11	BC1
	AN07,004	AN94,414,52	×	ALBA	10	BC1
	AN07,005	AN94,414,52	×	CLERY	10	BC1
B	AN07,006	AN00,239,55	×	Romina	8	BC2
	AN07,215	AN00,239,55	×	AN03,338,56	7	BC2
	AN07,216	AN00,239,55	×	CLERY	9	BC2
C	AN07,007	AN03,338,56	×	Romina	10	Intra-species
	AN07,009	CLERY	×	Romina	10	Intra-species

The corresponding parents and number of offspring evaluated for their fruit nutritional quality of the half-sib BC1 FVG, half-sib BC2 FVG and half-sib intra-species crossing. AN94,414,52 is a cross of the *Fragaria* × *ananassa* cultivar Don × *F. virginiana* ssp. *glauca* selection FVG 22 from USDA Corvallis germplasm repository (USA). AN00,239,55 (BC1) is an elite selection from the cross of selection AN94,414,52 (F1) × *F. × ananassa* selection 91,143,5. Romina and AN03,338,56 are elite selections from the Università Politecnica delle Marche breeding program, containing no wild germplasm.

These two intra-species cross populations also showed negative correlations between both of the color parameters, Chroma index and L* grade, and the fruit firmness and ACY, which means that the high color parameters correspond to a softer fruit with lower ACY (Table 4). Indeed, particularly for the fruits of the AN07,007 family, the significantly higher values of both of the color parameters correspond to significantly lower fruit firmness and ACY.

The PCA bi-plot of fruit nutritional parameters showed a clear distribution of the populations on the plot that highlights the selection AN07,007,55 as having the high values of the fruit nutritional parameters (TAC and TPH).

The PCA bi-plot of fruit weight, plant commercial production, and fruit nutritional parameters (TAC, TPH and ACY) for the offspring and parents of the intra-species cross combinations (Figure 8a) showed distinct distributions for the two populations (Figure 8b). Indeed, the offspring of AN07,007 were mainly positioned in the central-right-hand area of the plot, where the TPH and TAC vectors are located, while only AN07,007,57 is located in the lower right-hand quadrant. The offspring of AN07,009 are mainly located in the lower quadrant (Figure 8b), where the vectors of the fruit weight and commercial production variables are located (Figure 8a). The female parents, Clery and AN03,338,56, are located on the right-hand side of the plot (Figure 8b), where the TPH and TAC vectors are located (Figure 8a), while the common male parent, Romina, is located on the lower part of the plot, where the vectors for fruit weight, commercial production and ACY are located.

**Figure 8:** Principal component analysis. Bi-plot of the fruit weight, commercial production, TAC, TPH and ACY paraemters of the selections and the corresponding parents of the intra-species cross populations. Factor 1 and Factor 2 explain 65.95% of the data variation. a: Variable vector distributions; b: Case distributions. The seedlings reported in the PCA are identified only with the codes related to the cross combinations and the progressive seedling numbering.

The PCA bi-plot for fruit weight and commercial production combined with the sensorial parameters of SS content and TA (Figure 9a) distributes the offspring and parents widely in all four of the quadrants of the plot (Figure 9b). This distribution makes the different affinities of the two cross combinations towards the TA sensorial parameter clear. Indeed, the fruit of AN07,007 are located mainly towards the sensorial parameters vector TA (Figure 9b), while the fruit of the AN07,009 cross combination show a distribution that is mainly in the lower quadrants, on the opposite side of the TA vectors. From the distribution of the offspring, it can be noted that AN07,009,54, AN07,009,56 and AN07,009,60 are located in the lower left-hand quadrant, just in the opposite direction of the vectors that identify the TA variable, and also AN07,009,53, AN07,009,52 and AN07,009,51 are located on the lower part of the plot (Figure 9b), more oriented towards the SS content vector (Figure 9a). Half of the offspring of AN07,007, together with the female parents, AN03,338,56 and Clery, are located in the upper part of the plot (Figure 9b), between the vectors for the production variables and the fruit TA (Figure 9a). The offspring AN07,007,57 and AN07,009,57, together with the male parent (Romina), are located on the left-hand side of the plot (Figure 9b), where the production variables are located (Figure 9a). The selections AN07,007,53 and AN07,009,51, are located towards the SS content vector.

**Figure 9:** Principal component analysis. Bi-plot of the AWF, commercial production, SS conent and TA parameters of the selections and the corresponding parents of the intra-species cross populations. Factor 1 and Factor 2 explain 75.00% of the data variation. a: Variable vector distributions; b: Case distributions. The seedlings reported in the PCA are identified only with the codes related to the cross combinations and the progressive seedling numbering.

The PCA bi-plot for the fruit Chroma index, TPH and ACY parameters (Figure 10a) shows clear-cut distributions of the parents and offspring (Figure 10b). Indeed, the female parents together with most of the AN07,007 offspring are located on the left-hand side of the plot (Figure 10b), where the Chroma vector is located (Figure 10a), while the male parents and most of the AN07,009 offspring are on the right-hand side of the plot, which shows the separation between these two populations. The AN07,007 family is mainly located in the mid-upper part of the plot (Figure 10b), just on the opposite side of the TPH vector (Figure 10a).

**Figure 10:** Principal component analysis. Bi-plot of the Chroma, TPH and ACY parameters of the selections and the corresponding parents of the intra-species cross populations. Factor 1 and Factor 2 explain 90.87% of the data variation. a: Variable vector distributions; b: Case distributions. The seedlings reported in the PCA are identified only with the codes related to the cross combinations and the progressive seedling numbering.

The selection AN07,007,55 is located between the ACY and TPH vectors, while the selection AN07,009,56 is located towards the ACY vector, and the other offspring are not influenced by these variables (Figure 10b).

## Discussion

To date, strawberry breeding programs have been mainly focused on the improvement of agronomic and commercial traits [23], although more recently the major breeding targets have shifted more towards the sensorial and nutritional qualities of the strawberry fruit [24]–[25]. Very recent studies that have focused on the sensorial [26]–[27] and nutritional [4]–[7], [13]–[15], [24]–[25], [27] parameters in strawberry fruit have given more information and have considered further the concepts relating to their origins in plants and their importance for human health.

The major aim of the present study was to compare different breeding approaches to increase the narrow genetic base of the cultivated strawberry, and in particular, to increase the strawberry fruit sensorial and nutritional values. To achieve this, the contributions of *Fragaria virginiana* ssp. *glauca,* a wild octoploid strawberry, were tested in inter-species crosses and through subsequent back-cross cycles. The use of wild strawberry in this breeding program, which is aimed at producing new commercial varieties, is motivated by the need to increase the genetic variability of *Fragaria × ananassa* [28]–[29], because of the breeding selection process that has developed since the domestication of the first strawberry hybrids. The usefulness of FVG as an original source of fruit nutritional quality has already been reported [14]; however, long-term back-cross generations are necessary to provide new genotypes with high commercial value [5].

From the study of the inter-species back-cross populations, the offspring of BC1 and BC2 from FVG showed overall high fruit sensorial and nutritional qualities, as seen in the original F1 inter-species crosses [5]. These were combined with improvements in the other important commercial traits (mostly for fruit weight and commercial production), which were lost in the F1 lines. Indeed, the lack of association between the productivity and quality traits is well represented by the different PCA plots (Figures 2, 3, 5 and 6). These results highlight the independent genetic control of these important plant and fruit traits.

The use of FVG was also particularly efficient for the creation of greater variability, as seen with the production of a relatively high number of transgressive segregants. This result is considered to be particularly relevant in comparison with what was achieved from the *F. × ananassa* intra-species crosses included in the present study and in other studies [24]. Indeed, the FVG-derived populations had a higher number of new transgressive segregants, and also higher values for each of the sensorial and nutritional traits. This achievement is probably the result of an increased number of alleles that can interact epistatically [30], and also dominance/overdominance effects might have contributed to the presence of transgressive segregants for fruit quality [31].

The increase in fruit ACY is reflected phenotypically by the darker red coloration of the berry [24]. Fruit color is controlled at multiple levels that involve transcription factors and structural genes [32]–[33]. Quantitative trait loci for anthocyanin and fruit color have been evaluated for the *flavanone 3-hydroxylase, chalcone isomerase, flavonol synthetase* and *dihydroflavonol reductase* genes, which are involved in anthocyanin biosynthesis, but no gene co-location with fruit color or ACY was seen [25]. Improvements in the nutritional values in the BC1 and BC2 FVG populations, which were due in particular to increased ACY (Table 6), were associated with a decrease in the Chroma index. This was supported by the correlation matrix (Table 4), where these parameters were highly negatively correlated, both in the BC and intra-species offspring populations (Table 4) [24]. While for the intra-species populations, these were the only ones where a high negative correlation between colorimetric parameters and phenol content was confirmed [5], [15]. The PCA plots for the BC1 populations (Figure 4) show a high number of transgressive segregants for fruit color and ACY, while the BC2 populations do not show segregants. Hence, these data confirm the concept that fruit color is controlled by epistatic and dominance/overdominance effects [30]–[31], as seen for the nutritional compounds.

**Table 6:** Fruit sensorial and nutritional parameters of the BC1 and BC2 back-cross combinations and the intra-species cross combinations (evaluated in 2010 on clonal population of selected seedlings).

Type of Cross	SS content (°Brix)	TA (meq NaOH/100 g FW)	Firmness (g)	Chroma	L*	TAC(mmol TE/kg FW)	TPH(mg GA/kg FW)	ACY (mg PEL-3-GLU/kg FW)
BC1	9.40 a (0.15)	12.28 b (0.37)	336.00 b (8.26)	44.48 b (0.62)	34.24 b (0.36)	20.25 a (0.74)	1707.46 a (69.16)	464.16 a (19.09)
BC2	8.99 a (0.17)	13.55 a (0.42)	330.79 b (7.61)	42.67 b (0.66)	34.75 b (0.41)	21.42 a (1.09)	1708.72 ab (46.74)	484.34 a (21.1)
IS	8.45 b (0.18)	10.49 c (0.34)	381.77 a (11.47)	46.84 a (0.93)	37.54 a (0.66)	14.37 b (0.32)	1517.32 b (64.03)	353.97 b (25.69)

Data are means and standard errors (SE) of offspring selections for each cross combination type. Means followed by different letters are significantly different. SNK Test P≤0.05. IS, intra-species.

The importance of *F. virginiana*, and in particular ssp. *glauca*, for increases in pathogen resistance of the hybrid progenies was evaluated in a breeding program that was designed to widen the genetic base of the strawberry germplasm [22]. The BC1 and BC2 populations showed marked reductions in rotten fruit production in comparison to the *F. × ananassa* populations. This lower rotten fruit production was accompanied by a higher content of bioactive compounds, and specifically of anthocyanins and phenols, which have active roles in the protection of plants and fruit against pathogens [34]–[36]. Hence, the increases in the bioactive compounds in the BC1 and BC2 populations, and the data showing lower levels of rotten fruit production, can be considered as confirmation that the increased content of these bioactive compounds can have effects on increased tolerance to the major strawberry diseases [22]. Therefore, these achievements underline the importance of the wild genetic resources as sources of different important genes and the need for continued evaluation of back-cross generations for the creation of new genotypes with both improved nutritional compound content and disease resistance. Moreover, studies performed by Tulipani et al. [37] also showed that wild species can contribute to increases in not only interesting nutritional features in cultivated strawberry, but also in non-nutritional compounds, which might have implications for human consumption. From these findings, it is clear that intra-species crosses induce low increases in allergens contents, while the fruit from the F1 and BC1 selections had much higher contents of allergens.

In general, the performances of the BC1 and BC2 FVG populations can be further improved by additional back-cross generations, so as to be closer to the overall commercial quality that is required for any new commercial variety. By the third back-cross generation, the plant and fruit commercial standards can be very near to those requested for commercial cultivars [8].

The results for the *F. × ananassa* intra-species crosses show that there is a genetic background in the cultivated species that can induce an increase in the fruit sensorial and nutritional qualities. Even if these are of lower value in comparison with the FVG back-cross program, they are already combined with a high standard of commercial performance. However, this positive increase is strictly related to the genetic background of the selected parents. Indeed, the parents used in the cross combinations were chosen because they had already been identified as having high fruit nutritional quality in comparison with other cultivars [5], [12], [15].

### Conclusions

The present study has demonstrated that these two types of combination programs (inter-species back-crosses and intra-species crosses) can be used for the improvement of strawberry nutritional quality, although the success of the program is strictly related to the combining attitude of the different parents. For this reason, this type of experiment can be considered important for the production of new genotypes with improved sensorial and nutritional qualities, and for the identification of cultivars and selections that can perform in the same way as the most useful parents. These can be used in strawberry breeding programs that are aimed at the production of new improved varieties, for the better combination of the agronomic and overall fruit quality traits.

These evaluations carried out on the genetic pools that originated from the *F. virginiana* ssp. *glauca* inter-species back-cross and the *F. × ananassa* intra-species cross confirm the importance of using FVG, or genotypes with an FVG genetic background, in breeding programs aimed at increasing the fruit nutritional (TAC, TPH and ACY) and sensorial (SS content, TA, Chroma, L*, firmness) qualities. Indeed, both the BC1 and BC2 populations showed these characteristics, thus providing useful improvements in the fruit nutritional and sensorial qualities combined with agronomic standards that are closer to the those requested at the commercial level with respect to their respective FVG hybrid parents.

The results obtained in the present study show that two sequential back-crossing generations (BC1 and BC2) from an inter-species hybrid with a wild genotype of *F. virginiana* ssp. g*lauca* can improve sensorial and nutritional traits. These data confirm that at least two back-cross generations are needed to be close to the agronomic values requested at the commercial level [8].

This study has created new genotypes with the FVG genetic background introduced by inter-species crosses, thus increasing the genetic variability in cultivated strawberry, particularly for their specific nutritional traits [5]. This helps to counteract the narrow germplasm base that is used for breeding, which has caused deleterious effects of inbreeding and genetic vulnerability [27]. From our data, it is quite clear which parameters have to be increased in a back-crossing program. Fruit firmness, size, acidity and color are the main traits that can be recovered in the back-crossing generations. Clearly, the high positive values detected for some of the parameters in the F1 genotypes (TAC, polyphenols and folate) are reduced in the back-crossing generations, although they always remain higher than those in the commercial *F. × ananassa* genotypes. These findings suggest that controlled crosses of wild species with cultivated strawberry will contribute to introgression of interesting nutritional features; however, this can also lead to an increase in unfavorable compounds that might have health implications for humans, and that thus need specific evaluation.

Successive breeding studies using wild *Fragaria* octoploid species can introduce new genetic variability for nutritional, flavor and disease-resistance traits, and can contribute to our understanding of their heritability ratios and the hypothetical correlations with nutritional parameters [27]. Indeed, further studies on wild genotypes have evaluated the importance of FVG [22], and also of other wild genotypes with different ploidy levels [38]–[40], in terms of their flavor and resistance parameters, using gene expressions studies [41].

Improvements in sensorial and nutritional traits can also be achieved by the programming of *F. × ananassa* intra-species crosses and the production of progeny with productivity traits that are closer to those of the commercial cultivars, even if these improvements are fewer in number and quality with respect to the FVG back-cross populations.

## Materials and Methods

### Cross Combinations and Seedling Evaluations

A breeding program was carried out to obtain eight half-sib cross combinations originated using the following six different strawberry inter-species back-cross combinations and two intra-species cross combinations (Table 5, Figure 1):

- Three half-sib cross combinations originated as back-cross populations (BC1) with the F1 selection AN94,414,52, and an inter-species cross of *F. × ananassa* (Don) × *F. virginiana glauca* (FVG22) as the common parent;
- Three half-sib cross combinations originated as back-cross populations (BC2) with AN00,239,55, a BC1 selection derived from the back-crossing of selection F1 AN94,414,52 with 91,143,5 (*F. × ananassa* advanced selection) as the common parent;
- Two half-sib cross combinations originated by an intra-species cross with the selection Romina as the common parent.

Seedlings from all of these cross combinations were planted in 2008 in non-fumigated soil at the ‘P. Rosati’ University experimental farm, Agugliano (Ancona, Italy), and grown under open-field conditions using the plastic hill culture production system. For each cross combination of about 50 seedlings, seven to 11 elite seedlings were selected, based on a subjective phenotypic evaluation of the major plant vegetative and fruit sensorial traits, which was performed at the stage of fruit ripening. All of the seedlings of the different families were identified by code number, including AN as the Ancona site of the crossing, followed by 07 as the year of the crossing, with the code for the type of crossing, followed by progressive numbering (starting from 51) for each selected seedling. From this subjective selection, a total of 80 elite seedlings were identified and propagated by runners to create clonal population of the selected seedling. After the 2009 evaluation, 78 elite seedlings (two were lost) were planted as fresh plants in July 2009, in single plots of six plants each. They were then harvested and evaluated in May 2010, as selections from clonal population of selected seedlings.

This second evaluation was performed under the same open-field conditions in non-fumigated soil at the ‘P. Rosati’ University experimental farm, Agugliano (Ancona, Italy), again using the plastic hill culture production system. In the same field, under the same conditions, the corresponding parents of each of the cross combinations were also grown. Fruit samples of the fully red berries were harvested at the second, third and fourth main pickings. The evaluations took into account plant productivity (fruit weight and total plant production), and fruit nutritional (fruit TAC, phenols and ACY) and sensorial (fruit firmness, color, SS content and TA) parameters.

### Chemicals

The 99% methanol (ACS-ISO) for the analysis, and the bromothymol blue were purchased from Carlo Erba Reagenti (Milan, Italy). Folin-Ciocalteu’s reagent anhydrous, sodium carbonate, potassium chloride, sodium acetate, chloridric acid, glacial acetic acid, dihydrogen potassium phosphate, dipotassium hydrogen phosphate, 2,2′-azino-bis (3-ethylbenzothiazoline-6-sulphonic acid) diammonium salt (ABTS•+), 6-hydroxy-2,5,7,8-tetramethylchromane-2-carboxylic acid (Trolox), potassium persulfate, 3,4,5-trihydroxybenzoic acid (gallic acid), and sodium hydroxide, were purchased from Sigma-Aldrich (Milan, Italy).

### Strawberry Production Parameters

In 2010, the strawberry plant production was evaluated in the single plot of all of the selections at each harvest, by evaluating the following parameters:

- Total fruit production (g/plant).
- Commercial production: total weight (g/plant) of ripe fruit with a commercial diameter (Ø≤0.22 mm) and without injuries.
- Fruit weight: average weight (g) of 20 commercial fruits from each harvest.
- Undersized fruit: total weight (g/plant) of ripe fruits with diameter Ø ≥0.22 mm, without injuries.
- Misshapen fruit: total weight (g/plant) of misshapen fruits.
- Rotten fruit: total weight (g/plant) of rotten fruits.

### Strawberry Instrumental Sensorial Parameters

Fruit sensorial quality of the selections and the parents was analyzed on the harvesting day, at each harvest (2^nd^, 3^rd^, 4^th^), on 10 commercial fruits, taking in account the following parameters:

- SS content: determined using a hand-held refractometer (ATAGO), with results expressed as °Brix.
- TA: determined from 10 mL juice diluted with distilled water (1/2, v/v) and titrated with 0.1 N NaOH solution to pH 8.2, and expressed as mEQ of NaOH per 100 g fruit (fresh weight; FW).
- Fruit color: determined as the Chroma index using a Minolta Chromameter CR 400, for two sides of 10 sound, ripe, undamaged and uniform fruits. The instruments included three parameters L* (luminescence), a* (red tone), b* (yellow tone). The Chroma index was evaluated from a and b [(a*^2^+b*^2^)½], with a higher Chroma index representing pale fruit and a low Chroma index representing dark fruit.
- Fruit firmness: measured using a penetrometer 327 (Effegì, Ravenna, Italy), with the results expressed in g.

### Strawberry Nutritional Parameters

#### Fruit extraction method

From a pool of fruit for each genotype harvested in 2010 and stored at −20°C, 10 ripe commercial fruits were sampled, and from each fruit two slices from opposite sides were cut and milled into small pieces. Ten gram of this blend was weighed and placed into a tube for extraction with methanol (1∶4, fruit: methanol, w/w), including two subsequent steps. The first step consisted of homogenization with an Ultraturrax T25 homogenizer, for a fruit blend in 20 mL methanol (Janke and Kunkel, IKA Labortechnik, Staufen, Germany). The homogenized suspension was continuously agitated for 30 min in the dark. The suspension was centrifuged at 4,500×*g* for 10 min (Centrifuge Rotofix32, Hettich Zentrifugen, Tuttlingen, Germany), and the supernatant was collected and stored in three amber vials, of 1 mL each. For a more complete and extensive extraction, the pellet of the fruit was extracted a second time by adding another 20 mL methanol and repeating the procedure described above. The second supernatant was collected and added to the first one, always using 1 mL for each of the 3 amber vials per sample, and then stored at −20°C.

#### TAC

The fruit extract from each genotype was used to analyze the fruit TAC using the ABTS assay, according to a previously validated procedure [42]–[43]. ABTS is a chromogen and a colorless substance; it changes into its colored monocationic radical form (ABTS•+) with exposure to an oxidative agent. Addition of antioxidants reduces ABTS•+ into its colorless form. The extent of decolorization as a percentage of inhibition of ABTS•+ was determined as a function of the concentration and was calculated relative to the reactivity of Trolox, a water-soluble vitamin E analog. The antioxidant activity is expressed as mg Trolox equivalent per kg fresh pulp weight. The calibration was calculated as the linear regression from the dose-response of the Trolox standard.

#### TPH

The fruit TPH was evaluated on fruit extracts using the Folin-Ciocaltou’s reagent method [44], with gallic acid as the standard for the calibration curve. Briefly, a glass test-tube was filled with 7.0 mL water. Afterwards, 1 mL of the diluted sample (1∶20) was added, followed by the addition of 500 µL Folin-Ciocalteu-Reagent and vortexing. After 3 min, 1.5 mL sodium carbonate (0.53 mol/L) was added, and the tube was mixed once more and then stored in the dark for 60 min. The absorbance of the sample was measured at 760 nm after exactly 60 min. The data were calculated and expressed as mg gallic acid per kg fresh fruit, using a standard curve with the range of standard values of 10 to 50 mg gallic acid/L.

#### ACY

Total fruit ACY was measured on the fruit extracts using the pH differential shift method [45]. This assay is based on the anthocyanins characteristic of a change in intensity of hue depending on the pH shift. Briefly, the samples were diluted to a ratio of 1∶10 with potassium chloride (pH 1.00) and with sodium acetate (pH 4.50), and then the corresponding maximum absorbance for both of the solutions was measured at λ = 500 nm and at λ = 700 nm, respectively. The data were expressed as mg pelargonidin-3-glucoside (the anthocyanin more representative in strawberry) per kg fresh weight (mg Pel-3-Glu/kg FW).

### Experimental Trial and Statistical Analysis

In the 2010 harvest season, the fruit sensorial (SS content, TA, firmness, Chroma, L*) and nutritional (TAC, TPH, ACY) parameters were analyzed in triplicate for each clonal population of selected seedlings identified in 2009, and for their corresponding parents.

All of these data were subjected to the two-way nested analysis of variance, MANOVA test. The analysis of variance was performed for single cross types and single cross combinations as random effects. The data on fruit sensorial and nutritional parameters are reported as means±standard error (SE). Multiple comparisons were calculated according to the SNK test and were considered significant at p≤0.05.

Correlations among the sensorial (SS content, TA, firmness, Chroma, L*) and nutritional (TAC, TPH and ACY) parameters were analyzed using Pearson’s correlations. PCA was also used to evaluate the levels of association among the various production, sensorial and nutritional parameters of the selections that originated from the different cross combinations and their corresponding parents, calculated on a genotype-mean basis. Based on the theoretical arguments of PCA described by [46], the significant factor loading values ≥0.7 were used to identify the most important variables and observations in each dimension (PC). The factor loading values are the correlations of each variable with the PC. They are represented as vectors (positions) in the space represented by the axes of the PCA bi-plots (Figures 2a to 10a). In the graphs, the variables (Figures 2a to 10a) and observations (Figures 2b to 10b) that are closest to each other in the same geometric plane of the bi-plot are considered as interrelated, and as a result they are distant from the variables and observations to which they are not related, or are negatively related. The greater the distance of a vector from the origin of the axis, the higher the correlation of the variable with the PC represented in that dimension (axis). All of the analyses were performed using STATISTICA (Statsoft Inc., Tulsa, OK, USA).
